# Impact of Financing Constraints on Firm Performance: Moderating Effect Based on Firm Size

**DOI:** 10.1155/2022/1954164

**Published:** 2022-08-12

**Authors:** Yonghong Yao, Jing Feng, Qiaowen Yang

**Affiliations:** Accounting School, Guangzhou Huashang College, Guangzhou 511300, China

## Abstract

This paper selects the relevant data of Shanghai and Shenzhen NG listed companies from 2016 to 2020 as the research object. By drawing on relevant research results at home and abroad, the variable KZ is used to measure the degree of corporate financing constraints, and the variable Tobin Q is used to measure corporate performance. The test draws the following conclusions: financing constraints are conducive to improving corporate performance. The reason is that the higher the degree of corporate financing constraints is, the more cautious the managers are in the use of funds, and the company managers can formulate more scientific management strategies, so as to improve corporate performance. Through further research, it is found that, with the expansion of the scale of the enterprise, the degree of financing constraints has less negative impact on the performance of the enterprise. Performance has a positive impact. According to the above conclusions, the government should improve the financial market system, build a multilevel capital market, and fundamentally ease the financing constraints of enterprises, to develop and improve self-management.

## 1. Introduction

The relationship between financing constraints and firm performance is an important issue in the field of financing; however, academic research on the relationship between the two has drawn different conclusions. With the increasingly fierce market competition, many enterprises blindly pursue economic interests while ignoring other problems caused by financing. As a profit-oriented economic unit, there is no doubt that enterprises pursue economic interests, while ignoring the existence of long-term interests. Through financing activities, enterprises can improve corporate performance and further promote the sustainable development of enterprises, but the relationship between financing constraints and corporate performance is not one-way, but mutual influence and mutual promotion. The size of the enterprise has a certain influence on the financing constraints. For example, the larger enterprises have stronger economic strength, which inhibits the financing constraints. Compared with the smaller enterprises, the smaller the financing constraints of the large enterprises, the higher the financing constraints. At the same time, for enterprises of different sizes, the degree of the relationship between financing constraints and performance will also be different, so the size of the enterprise has a certain moderating effect on financing constraints and corporate performance. This paper takes the data of Shanghai and Shenzhen A-share listed companies from 2016 to 2020 as the research sample, draws on relevant research results at home and abroad, uses the variable KZ to represent the degree of corporate financing constraints, uses Tobin's Q to measure corporate performance, and empirically tests financing constraints. With the impact on enterprise performance, and through further research, analyze the adjustment effect of enterprise scale on financing constraints and enterprise performance, and provide reference for the government and enterprises to formulate relevant policies by improving relevant research.

## 2. Literature Review

Based on the research purpose of this paper, through the selection, comparison, classification, and analysis of relevant literature, starting from the relationship between financing constraints and corporate performance, and the adjustment effect of corporate size on financing constraints and corporate performance, the relevant literature is analyzed. The specific content is as follows.

### 2.1. The Relationship between Financing Constraints and Firm Performance

Since financing constraints have a significant impact on corporate performance, it will have a greater impact on corporate business decisions. By reading the relevant literature, it is found that the researchers' research on related issues is mainly based on the financing priority theory, MM theory, information asymmetry theory, and agency theory. There are several studies on the relationship between financing constraints and corporate performance. Different conclusions are discussed below.

Badia and Slootmaekers [1] concluded through empirical research that if an enterprise is constrained by financing in the process of financing, the amount of funds in the company will be easily limited, which will prompt corporate personnel and encourage managers to use funds, improve the efficiency of capital use, and further improve corporate performance. Chen [2] also found through research that, in order to complete their tasks, business operators with financing constraints must select projects with high returns from limited funds to operate in order to use funds efficiently, thereby helping to improve enterprises performance. He [3] used the data of listed companies on the Growth Enterprise Market and concluded through empirical research that the higher the financing constraint, the higher the corporate performance, and the two are positively correlated. Qiu and Wang [4] found through research that higher financing constraints can promote the positive effect of R&D investment on corporate performance. However, some scholars have come to the opposite conclusion. Hovakimian and Titman [5] believe that the financing constraints of enterprises are not conducive to the improvement of technology and productivity and thus will have a negative impact on enterprise performance. Ni [6] found that financing difficulties are one of the important reasons hindering the development of Chinese enterprises. The survival and development of enterprises need financial support, but due to the existence of financing constraints, the R&D needs of enterprises cannot be met, thus inhibiting enterprises performance improvement. Xu [7] conducted an empirical study on the SMEs listed on the Shenzhen Stock Exchange from 2011 to 2015 and found that the financing constraints of SMEs have a strong negative impact on corporate performance. There are also studies show that financing constraints are not significantly related to corporate performance. Gu et al. [8] found that financing constraint indicators in different dimensions have different effects on corporate performance by constructing financing constraint indicators. The effect was not significant.

### 2.2. The Relationship between Firm Size and Financing Constraints

In order to study the impact of firm size on financing constraints more deeply, researchers have explored and analyzed it from different perspectives. Some researchers believe that the increase of enterprise scale can alleviate the problem of financing constraints. Luo [9] studied the relationship between investment expenditure and internal funds of Japanese listed companies and believed that the degree of financing constraints suffered by enterprises in the external capital market varies with the size of the enterprise. Some scholars believe that the increase of enterprise scale will intensify financing constraints. Vogt [10] and Athey and Laumas [11] have found through empirical research that if the enterprise scale gradually increases, the sensitivity of investment current flow will gradually decrease, which will lead to financing constraints. Kadapakarm et al. [12], Ma and Dong [13], and other studies believe that, with the increase of the scale of enterprises, the degree of information disclosure is also increasing, and the degree of information asymmetry between banks will increase due to low information transparency. To a certain extent, it has increased the pressure on enterprises to obtain financing from banks.

### 2.3. Research on the Relationship between Firm Size and Firm Performance

Although domestic and foreign researchers have conducted a lot of research on the relationship between firm size and firm performance, they have not yet reached a consistent conclusion. Fan and Zhou [14], Mu and Zhang [15], Lu [16], and others concluded through empirical research that firm size has a significant negative impact on firm performance. However, Porter [17] found through empirical research that once an enterprise achieves economies of scale, it can effectively improve enterprise performance and promote enterprise development. Ling and Hu [18] also obtained similar results through empirical research; that is, the expansion of the scale of strategic emerging companies is conducive to improving corporate performance. In addition, a small number of researchers have come to the conclusion that there is no linear correlation between enterprise scale and enterprise performance. Yao [19] selected the relevant data of A-share listed companies from 2009 to 2018 as research samples and studied the relationship between enterprise scale and enterprise performance and correlation with performance and finally concluded that there is a significant inverted U-shaped relationship between firm size and firm performance.

### 2.4. Literature Review

The conclusions of the above researchers are different. The possible reason is that the researcher's research background, the characteristics of the selected samples, and the index measurement methods are different. So far, researchers have more understanding of the relationship between enterprise scale, financing constraints, and corporate performance but less research on the moderating relationship between corporate financing constraints and financial performance from an empirical perspective [20–25]. Therefore, this paper will focus on the basis of previous research, further explore the correlation between financing constraints and corporate performance, and add corporate size as a moderating variable between financing constraints and corporate performance, focusing on the moderating effect of corporate size on financing constraints and corporate performance to supplement and complete relevant research.

## 3. Theoretical Analysis and Research Assumptions

### 3.1. The Impact of Financing Constraints on Firm Performance

There are different conclusions about the impact of financing constraints on corporate performance. Generally speaking, if the financing constraints are higher, the improvement of corporate performance will be inhibited; that is, financing constraints have a significant negative impact on corporate performance. However, some people believe that the higher the financing constraint is, the higher the corporate performance will be; that is, the financing constraint has a significant positive impact on corporate performance. According to the theory of information asymmetry, in an imperfect market, the information held by both parties is not exactly the same, and those with poor information pay higher costs than those with abundant information. The principal-agent theory holds that the higher the financing constraints of the enterprise, the higher the opportunity cost, which makes the management more cautious in the investment decision, so as to improve the efficiency of capital use and then improve the performance of the enterprise. This paper argues that, under normal circumstances, there are certain restrictions for companies to raise funds. The greater the pressure on R&D funds, the greater the investment risk and financial risk. Because managers cannot bear the financial risks brought by decision failure, they will pay more attention to the efficiency of the use of funds. Therefore, due to the existence of financing constraints, it will help the improvement of corporate performance. Based on the above discussion, this paper proposes the following assumptions.

**Hypothesis 1 .**

Financing constraints have a positive impact on firm performance.

### 3.2. The Moderating Effect of Firm Size on Financing Constraints and Firm Performance

The size of an enterprise has a great influence on its operating efficiency, operating results, financial income, and expenditure and reputation, and the correlation between various factors is very large. Usually, large-scale enterprises have sufficient working capital, which leads to relatively stable operations. When faced with financial pressure, they tend to adopt a parallel strategy of multiple financing methods, so that they are less constrained by financing, which in turn makes its financing costs relatively low. At the same time, larger enterprises can gain economies of scale in R&D, which will further improve their performance. On the contrary, small-scale enterprises need less capital and less financing channels, so their financing constraints are relatively high, and their financing costs will increase relatively. In addition, knowledge has the characteristics of public goods, and the cost of using knowledge is relatively lower for large-scale enterprises than small enterprises. Therefore, large-scale enterprises have higher returns on large-scale investment than small-scale enterprises. In summary, this paper proposes the following assumptions.

**Hypothesis 2 .**

Firm size has a positive moderating effect on financing constraints and firm performance.

## 4. Study Design

### 4.1. Sample Selection

Considering the availability and comprehensiveness of data, this paper takes the relevant data of Shanghai and Shenzhen A-share listed companies from 2016 to 2020 as the research sample. The data is mainly from the CSMAR and WIND databases, and the following data processing is mainly carried out: (1) the PT, ST, and ^*∗*^ST and other Ts in the sample are excluded; (2) exclude financial listed companies from the sample; (3) exclude companies with missing data in the sample—annual observation value. In addition, this paper also shortens the row of continuous variables to avoid the influence of extreme values on the regression results. After the above processing, this article finally got 3013 sample companies. Among them, EXCEL software was used for data processing, and STATA15.0 was used for data processing.

### 4.2. Variable Definition

#### 4.2.1. Enterprise Performance

This paper uses Tobin's Q to measure firm performance. Tobin's Q is easy to obtain in the database and has both theoretical and practical operability and can be used to represent enterprise performance.

#### 4.2.2. Degree of Financing Constraints

Some key indicators, such as operating net cash flow, debt level, cash holdings, and enterprise growth can indirectly reflect the degree of financing constraints of enterprises [21]. The researchers regressed these factors to construct the KZ index. The index is mainly used to measure the corresponding degree of financing constraints of enterprises. Since then, this method has been widely used in the study of financing constraints related issues. This paper draws on the research ideas of Kaplan and Zingales [26] and the research methods of Tan and Xia [27] and Wei [28] and uses the KZ index as an indicator to measure financing constraints, the higher the degree of financing constraints faced by the company.

#### 4.2.3. Classification of Enterprise Size

According to the enterprise scale classification method in the “Small and Medium Enterprises Promotion Law of the People's Republic of China,” the logarithm of total assets is used as a measure of enterprise scale. If ln (SIZE) ≥ 23.05, it is a large enterprise; For medium-sized enterprises; if (SIZE) < 20.7, it is a small enterprise.

#### 4.2.4. Control Variable Selection

This paper draws on the existing relevant research literature and selects the following variables as the control variables of this paper: (1) Age of the enterprise (AGE): The general theory holds that the longer an enterprise has been established, the more operational experience it can accumulate, and the enterprise will have abundant financing channels, which will have a better impact on enterprise performance; (2) assets-liability ratio (LEV): The asset-liability ratio is used to measure the solvency of an enterprise, and it is also used to reflect the capital structure of the enterprise. When the asset-liability ratio is greater than 100%, it indicates that the company is insolvent. The theoretical data of the critical point of the asset-liability ratio is 50%. If it is obviously lower than 50%, the risk will be small, the use of external funds will be small, and the development will be relatively slow; if it is close to or higher than 50%, the risk factor will be large, but the use of external funds will lead to development relatively fast; (3) net assets per share (BPS): The net asset value per share reflects the company's net asset value represented by each share and is an important basis for supporting the stock market price. The larger the net asset value per share, the stronger the wealth per share of the company, and the stronger the ability to generate profits and resist the influence of external factors. The definitions of related variables are shown in Table 1.

### 4.3. Model Design

This paper designs the following model to test the hypothesis:

(1) $$\begin{array}{c} \left(1\right)\text{Tobin's}{\text{Q}}_{\text{it}}=\beta_{\text{0}}+\beta_{1}{\text{KZ}}_{\text{it}}+\beta_{2}{\text{AGE}}_{\text{it}}+\beta_{3}{\text{LEV}}_{\text{it}}+\beta_{4}{\text{BPS}}_{\text{it}}+\varepsilon ,\\ \text{Tobin's}{\text{Q}}_{\text{it}}=\beta_{0}+\beta_{1}{\text{KZ}}_{\text{it}}+\beta_{2}{\text{SIZE}}_{\text{it}}+\beta_{3}{\text{AGE}}_{\text{it}}+\beta_{4}{\text{LEV}}_{\text{it}}+\beta_{5}{\text{BPS}}_{\text{it}}+\varepsilon ,\\ \text{Tobin's}{\text{Q}}_{\text{it}}=\beta_{0}+\beta_{1}{\text{KZ}}_{\text{it}}+\beta_{2}{\text{SIZE}}_{\text{it}}*\beta_{3}{\text{AGE}}_{\text{it}}+\beta_{4}{\text{LEV}}_{\text{it}}+\beta_{5}{\text{BPS}}_{\text{it}}+\varepsilon . \end{array}$$

In the model, *β*0 is a constant term, *β*_*i*_ (*i* = 1, 2, 3, 4, 5) is a regression coefficient, *ε* is a random error term, and the meanings of other variables are shown in Table 1.

Hypothesis 1 is tested by observing the positive or negative of the regression coefficient *β*_1_ in the above model (1), and Hypothesis 2 is tested by using the hierarchical regression analysis method in model (2), that is, by observing model (1), and the change of R2 in model (2) can be used to judge whether there is a moderating effect on the scale of the enterprise, and the positive or negative of the moderating effect can be judged by observing the correlation coefficient *β*_2_ of the interaction term (SIZE _it_^*∗*^KZ _it_) in model (2).

## 5. Empirical Results

### 5.1. Descriptive Statistics

In order to better understand the distribution of the data, this paper firstly conducts descriptive statistics on the sample data. The specific results are shown in Table 2.

Table 2 shows the descriptive statistics of the variables. The mean of Tobin's Q is 2.1246 and the standard deviation is 2.0444, which is less than the mean. The results are in line with expectations, indicating that the overall data is ideal and there are no extreme outliers. The standard deviation of KZ is 2.212398, the minimum value is −6.1759, and the maximum value is 5.4558. The above statistical analysis results show that the degree of financing constraints between Shanghai and Shenzhen A-share listed companies is relatively different. SIZE is a measure of company size, with a mean value of 22.4153, indicating that most of the sample data are medium-sized enterprises, and the standard deviation is 5.8840, which is less than the average value, indicating that the overall difference in enterprise size is relatively small, but there are still some large-scale enterprises, or very small extreme value businesses. The control variables AGE, LEV, and BPS were observed and it was found that their standard deviations were all smaller than the mean value, indicating that the analysis conditions were met [29]. Overall, the data are ideal and can meet the further analysis needs of this paper.

### 5.2. Correlation Test

The test belongs to the Pearson correlation test, and its function is to simply consider the relationship between variables related relationship. The test results are shown in Table 3.

It can be seen from Table 3 that the correlation coefficients before the variables are all less than 0.7, indicating that the degree of correlation between the variables is low, which further indicates that the selection of variables in this paper is reasonable and meets the needs of model analysis. In the table, the correlation coefficient between financing constraint KZ and Tobin's Q is -0.0910, which is significant at the 1% level. However, further regression analysis is required for the specific research conclusions. The correlation coefficient between the asset-liability ratio LEV and Tobin's Q is −0.4069, the correlation coefficient between the asset-liability ratio LEV and the financing constraint KZ is 0.5643, and both are significantly correlated at the 1% level. Although the asset-liability ratio LEV has a strong correlation with Tobin's Q and KZ, it does not exceed the critical value of 0.7, which shows that corporate performance and financing constraints are strongly dependent on the asset-liability ratio to a certain extent. Therefore, in order to avoid the influence of collinearity between variables, this paper conducts multicollinearity test (VIF test) before regression analysis, in order to avoid the problem of false regression.

### 5.3. Regression Results and Analysis

#### 5.3.1. Regression Analysis of Financing Constraints and Firm Performance

This part mainly uses model (1) to perform regression analysis on the correlation between financing constraints and corporate performance. First, before the regression of model (1), the variance inflation factor (VIF) of the relevant variables in the model is estimated to test the multicollinearity problem, as shown in Table 4.

In general, if the variance inflation factor (VIF) > 10, it means that there is a multicollinearity problem in the model. From Table 4, it can be seen that the VIF statistic is between 1 and 10, and it is considered that the variables selected in this paper are no multicollinearity, so it can be directly added to the regression model. The regression results are shown in Table 5.

Observing Table 5, it is found that the regression coefficient of financing constraint KZ is 0.1517, and it is significantly positive at the level of 1%. The empirical research results show that financing constraints have a significant positive impact on corporate performance. Hypothesis 1 of this paper is verified, so for enterprises with higher financing constraints, enterprise managers will be more cautious in the use of funds and strictly control all aspects of production and sales above the existing development level to ensure that enterprise funds are used reasonably and make enterprise performance be effectively improved. And compared with the previous correlation analysis results, it is found that the control variable selection in this paper is effective.

#### 5.3.2. Regression Analysis of the Adjustment Effect of Enterprise Scale on Financing Constraints and Enterprise Performance

This part mainly conducts regression analysis on the moderating effect of enterprise size. Before regression analysis of model (2), the variance inflation factor (VIF) of relevant variables in model (2) is estimated first. The specific results are shown in Table 6.

It can be seen from Table 6 that if the VIF statistic is between 1 and 10, it is considered that there is no multicollinearity among the variables selected in this paper, so the regression model can be directly added, and in the regression analysis, the adjustment variable and the independent variables are decentralized. The regression results are shown in Table 7.

By observing Table 7, it is found that, for adjusting the scale of the enterprise, in model (1) without the SIZE^*∗*^KZ interaction term, the R2 of the model is 0.1036, and in the model (2) with the SIZE^*∗*^KZ interaction term added, the *R* ^2^ of the model is 0.1049. By comparing the adjusted *R* ^2^ of model (1) and model (2), it is found that the *R* ^2^ of model (2) has increased compared with model (1). Therefore, the moderating effect of firm size on financing constraints and firm performance exists. Further analyze the specific embodiment of the adjustment effect of enterprise scale. By observing Table 7, it is found that the SIZE^*∗*^KZ interaction term regression coefficient is 0.0133 > 0, and it is significantly positive at the 5% level. Therefore, with the expansion of the enterprise scale, the positive effect of financing constraints on enterprise performance is not weakened but further strengthened. Hypothesis 2 is verified.

## 6. Research Conclusions and Policy Recommendations

### 6.1. Research Conclusions

This paper uses the data of A-share listed companies in Shanghai and Shenzhen from 2016 to 2020 as the research sample and draws on the existing related research at home and abroad. To measure the size of enterprises, we empirically test the impact of financing constraints on corporate performance and the moderating effect of corporate size on financing constraints and corporate performance. The following two conclusions are drawn from the empirical research:

1. Financing constraints are conducive to improving corporate performance. Under the existing market economy conditions, companies with higher financing constraints will adopt relatively conservative development strategies in the development process, such as using the company's internal funds more cautiously, in preparation for new development opportunities in the future. There are enough funds to invest, thereby enhancing the comprehensive competitiveness of the company; in the face of greater financing constraints, company managers can formulate more scientific management strategies, optimize personnel allocation, reduce expenses, and make the company's funds rationally used. In turn, it will increase the overall operational efficiency of the enterprise, thereby improving the performance of the enterprise.
2. The larger the enterprise scale, the smaller the negative impact of the degree of financing constraints on enterprise performance. Although the financing constraints mentioned above are conducive to improving corporate performance, this is only in the short term. In the long run, the existence of financing constraints will force companies to abandon some favorable investment projects, thus making them stagnant, and market competition force is reduced. With the continuous expansion of the scale of enterprises, when faced with financing constraints, enterprises will adopt a variety of financing methods to relieve capital pressure and adopt various financing methods to reduce financing costs at the same time. Therefore, with the expansion of enterprise scale, its fundswhich has a positive impact on corporate performance.

### 6.2. Policy Recommendations

1. Improve the financial market system and enhance the hierarchy of the capital market. Through empirical research, it is found that the current financing methods of Chinese enterprises are relatively simple, and most enterprises are forced to occupy more free funds, which will make enterprises miss a lot of investment opportunities. Development faltered. In response to this situation, the government should further improve the financial market system, strengthen the supervision of the financial market, enhance the hierarchy of the capital market, alleviate the financing constraints of enterprises from the root, and strengthen the supervision of the use of external funds of enterprises to increase funds efficiency of use.
2. Enterprises should expand their own scale and seek diversified development. Larger enterprises have sufficient working capital, which leads to their relatively stable operations. When facing financial pressure, they tend to adopt a strategy of multiple financing methods in parallel, so that they are less constrained by financing, and thus make their financing cost be relatively low. Small-scale enterprises need less capital and have relatively few financing channels, so their financing constraints are relatively high, and financing costs will increase relatively. Therefore, appropriately expanding the scale of enterprises can give full play to the advantages of economies of scale. At the same time of scale, implementing diversified management of enterprises, taking strategic investment, and expanding the scale of enterprises through mergers and acquisitions, etc., can achieve large-scale development of enterprises.

## Figures and Tables

**Table 1:** Variable definition table.

Variable type	Variable abbreviation	Variable definitions
Explained variable	Tobin's Q	Measure business performance
Explanatory variables	KZ	Measure the degree of corporate financing constraints
Moderator	SIZE	Company size, log total assets: LN (total assets)
Control variable	AGE	The age of the enterprise, according to the time of establishment of the enterprise, calculate the time span of the year under study
	LEV	Asset-liability ratio = total liabilities at the end of the period/total assets at the end of the period
	BPS	Net assets per share = shareholders' equity/total share capital

**Table 2:** Descriptive statistics of variables.

Variable name	Observations	Mean	Standard deviation	Minimum value	Maximum value
Tobin's Q	10172	2.1246	2.0444	0.1377	11.9248
KZ	10172	0.5047	2.2123	-6.1759	5.4558
SIZE	10172	22.415	1.441	19.768	27.318
AGE	10172	19.053	5.884	4	52.67
LEV	10172	0.4323	0.2029	0.0643	0.9088
BPS	10172	5.4270	3.7565	0.3785	23.3642

**Table 3:** Variable correlation coefficient table.

	Tobin's Q	KZ	SIZE	AGE	LEV	BPS
Tobin's Q	1
KZ	−0.0910^∗∗∗^	1
SIZE	−0.0211^∗∗^	0.0238^∗∗∗^	1
AGE	−0.0346^∗∗∗^	−0.0169^*∗*^	0.2022^∗∗∗^	1
LEV	−0.4069^∗∗∗^	0.5643^∗∗∗^	0.0628^∗∗∗^	0.0055	1
BPS	0.0187^*∗*^	−0.0136	0.0629^∗∗∗^	0.1026^∗∗∗^	0.0024	1

*Note*. ^∗∗∗^, ^∗∗^, and ^*∗*^ are significant at the 1%, 5%, and 10% levels, respectively.

**Table 4:** VIF statistics of financing constraints and firm performance.

Variable	Model (1)
KZ	1.47
AGE	1.47
LEV	1.01
BPS	1.01

**Table 5:** Regression results of financing constraints and firm performance.

Variable	Model (1)
*β*_0_	5.7713^∗∗∗^
KZ	0.1517^∗∗∗^
AGE	−0.0905^∗∗∗^
LEV	−4.8085^∗∗∗^
BPS	0.0218^∗∗∗^
*R* ^2^	0.11

*Note*. ^∗∗∗^, ^∗∗^, ^*∗*^ are significant at the 1%, 5%, and 10% levels, respectively.

**Table 6:** VIF statistics of the adjustment effect of firm size.

Variable	Model (2)
KZ	1.47
SIZE	1.05
AGE	1.05
LEV	1.47
BPS	1.01

**Table 7:** The regression results of the adjustment effect of enterprise size.

Variable	Model (2)	
	(1)	(2)
*β*_0_	5.7157^∗∗∗^	0.2946^∗∗∗^
KZ	0.1519^∗∗∗^	0.1513^∗∗∗^
SIZE	−0.0918 ^∗∗∗^	−0.0924^∗∗∗^
SIZE^*∗*^KZ		0.0133^∗∗∗^
AGE	−0.0846^∗∗∗^	−0.0850^∗∗∗^
LEV	−4.7843^∗∗∗^	−4.7804^∗∗∗^
BPS	0.0226^∗∗∗^	0.0228^∗∗∗^
*R* ^2^	0.1036	0.1049

*Note.* ^∗∗∗^, ^∗∗^, ^*∗*^ are significant at the 1%, 5%, and 10% levels, respectively.

## Data Availability

The data used to support the findings of this study are available from the corresponding author upon request.
